This article has been retracted.

# Survivin knockdown alleviates pathological hydrostatic pressure-induced bladder smooth muscle cell dysfunction and BOO-induced bladder remodeling *via* autophagy

**DOI:** 10.3389/fcell.2022.999547

**Published:** 2022-10-28

**Authors:** Guo Chen, Shuang Chen, Xingpeng Di, Shengyin He, Yugao Liu, Rui Qu, Yi Luo, Yuebai Liu, Luo Yang

**Affiliations:** ^1^ Department of Urology, West China School of Public Health and West China Fourth Hospital, Sichuan University, Chengdu, China; ^2^ Laboratory of Reconstructive Urology, West China Hospital, Institute of Urology, Sichuan University, Chengdu, China; ^3^ Department of Education and Training, Sichuan Cancer Hospital, Chengdu, China

**Keywords:** survivin, autophagy, bladder smooth muscle cell, bladder outlet obstruction, bladder remodeling

## Abstract

**Aim:** Bladder outlet obstruction (BOO) leads to bladder wall remodeling accompanying the progression from inflammation to fibrosis where pathological hydrostatic pressure (HP)-induced alteration of bladder smooth muscle cells (BSMCs) hypertrophic and excessive extracellular matrix (ECM) deposition play a pivotal role. Recently, we have predicted survivin (BIRC5) as a potential hub gene that might be critical during bladder fibrosis by bioinformatics analyses from rat BOO bladder, but its function during BOO progression remains unknown. Here, we investigated the role of survivin protein on bladder dysfunction of BOO both *in vitro* and *in vivo*.

**Methods:** Sprague-Dawley female rats were divided into three groups: control group, BOO group, and BOO followed by the treatment with YM155 group. Bladder morphology and function were evaluated by Masson staining and urodynamic testing. To elucidate the underlying mechanism, hBSMCs were subjected to pathological HP of 200 cm H_2_O and co-cultured with the presence or absence of survivin siRNA and/or autophagy inhibitor 3-MA. Autophagy was evaluated by the detection of Beclin1 and LC3B-II expression, proliferation was conducted by the EdU analysis and PCNA expression, and fibrosis was assessed by the examination of Col 1 and Fn expression.

**Results:** BOO led to a gradual alteration of hypertrophy and fibrosis of the bladder, and subsequently induced bladder dysfunction accompanied by increased survivin expression, while these histological and function changes were attenuated by the treatment with YM155. HP significantly increased survivin expression, upregulated Col1 and Fn expression, enhanced proliferation, and downregulated autophagy markers, but these changes were partially abolished by survivin siRNA treatment, which was consistent with the results of the BOO rat experiment. In addition, the anti-fibrotic and anti-proliferative effects of the survivin siRNA treatment on hBSMCs were diminished after the inhibition of autophagy by the treatment with 3-MA.

**Conclusion:** In summary, the upregulation of survivin increased cell proliferation and fibrotic protein expression of hBSMC and drove the onset of bladder remodeling through autophagy during BOO. Targeting survivin in pathological hBSMCs could be a promising way to anti-fibrotic therapeutic approach in bladder remodeling secondary to BOO.

## Introduction

Bladder outlet obstruction (BOO) is characterized by gradually increased intravesical hydrostatic pressure and low flow micturition pattern, is a prevalent condition among aging males that is primarily caused by benign prostatic hyperplasia (BPH) (Capolicchio et al., 2001; Metcalfe et al., 2010; Chen et al., 2012; Komninos and Mitsogiannis 2014). Given the irreversible bladder remodeling, late-stage BOO characterized by bladder decompensation has poor success rates in improving the voiding symptoms even after surgical treatments, which seriously affects the quality of life of patients and their partners (Komninos and Mitsogiannis 2014). Understanding the underlying mechanisms of obstruction to fibrosis may contribute to identifying new targets for pharmaceutical intervention and ensure that patients who live with a degree of obstruction never progress to the end stages of bladder dysfunction.

As shown in previous studies, the role of cytokines including alpha-blockers, antimuscarinics, and *β*-Adrenergic receptors during BOO has been well-established (Dale et al., 2014; Gumrah et al., 2017; Yamada et al., 2018). In addition, TGF-β signaling could stimulate fibrotic changes in BSMCs after BOO, and miR-133 could modulate TGF-β-induced BSMC phenotypic changes by targeting CTGF (Duan et al., 2015). Platelet-derived growth factor could induce the proliferation of BSMC and basic fibroblast growth factor could upregulate Col3 and induce the proliferation of BSMC (Imamura et al., 2007; Preis et al., 2015). Hypoxia also affected the BSMC fibrosis, and miR-101 protected hypoxia-induced fibrosis by attenuating TGF-β-smad2/3 signaling (Wang et al., 2019). YAP inhibitor verteporfin improved the pathophysiologic changes of BSMC through the regulation of DNA methylation (Sidler et al., 2018). Moreover, increasing evidence indicated that mechanical stimuli contribute to bladder growth and development; while abnormal mechanical conditions secondary to BOO result in detrusor smooth muscle hypertrophy and extracellular matrix (ECM) accumulation (Ito et al., 2021). Our laboratory demonstrated that intravesical hydrostatic pressure triggered multiple signaling pathways including ERK, NF-κB, PI3K/SGK1, AMPK/mTOR, and so on that were involved in inflammation, dedifferentiation, and fibrosis (Chen et al., 2012; Chen et al., 2015; Liang et al., 2017; Chen et al., 2020a). But the mechano-regulatory processes during BOO remain unknown.

Survivin is the smallest member of the inhibitor of apoptosis protein (IAP) family discovered in 1997 (Li et al., 2021). Recently, emerging evidence has suggested that survivin was highly expressed in most tumor tissues and fibrotic diseases, and its expression was associated with a diverse array of cellular pathological and physiological processes such as differentiation, proliferation, and invasion during scarring, liver fibrosis, and vascular remodeling (Fan et al., 2015; Wang et al., 2018; Sharma et al., 2021; Ye et al., 2022). Interestingly, our previous study has predicted that survivin was significantly associated with the fibrotic stage of BOO (Di et al., 2022). However, its effects during bladder remodeling remain unclear and require further investigation.

Autophagy is a highly regulated catabolic process that maintains cellular homeostasis in response to various damaged, defective, or unwanted stimuli (Geir et al., 2005; Li et al., 2016; Daniel et al., 2018; Nam et al., 2019). Increasing evidence suggests that autophagy is closely related the bladder remodeling secondary to BOO due to its double-edged sword role in pro-cell survival and the pro-cell death properties (Chen et al., 2021). Our previous study has demonstrated that autophagy regulated the biological function of BSMCs under HP (Chen et al., 2020b). The emerging data indicated that survivin negatively modulated autophagy levels in various diseases, which piqued our interest in exploring whether the survivin has a similar role in the bladder remodeling of BOO (Ding et al., 2015; Pavel et al., 2018). We hypothesize that survivin plays a crucial role in the pathological process of bladder remodeling during BOO. In the present study, BOO rats were administered with survivin inhibitor YM155 to demonstrate the effect of survivin. To examine its possible underlying mechanism, cells were subject to HP to simulate the mechanical obstruction microenvironment of BOO. The mechanism in this pathological process provided new ideas for the prevention and targeted therapy of bladder remodeling after BOO.

## Materials and methods

### Rat bladder outlet obstruction model and experimental design

All animal experiments were reviewed and approved by the West China Hospital Committee on Animal Care. Female rats (220–250 g) underwent surgical operation for the establishment of BOO was similar to our previous study (Liu et al., 2017). The sham-operated group underwent the same procedure but without urethral ligation. BOO rats in the experimental group were administered with survivin inhibitor YM155. The control group was treated with saline. BOO rats were given by gavage orally administered with 10 mg/kg YM155 or saline once other days from the third day after the operation for 6 weeks. After 6 weeks, the urodynamic characteristics were detected. Subsequently, rats were humanely euthanized for the detection of bladder weight, bladder structure, bladder fibrosis, and mucosa-removed for WB.

### Urodynamics

Cystometry was performed to evaluate the urodynamic parameters as previously described. Briefly, rats were anesthetized and a 25 G needle connecting to a polyethylene catheter was inserted and fixed in the dome of the bladder. Cystometry was performed through the continuous saline infusion at a rate of 2.4 ml/h. The micturition pressure, baseline pressure, threshold pressure, and micturition interval were recorded to evaluate bladder function.

### Histology and immunohistochemistry

After the end of the cystometry, bladders were excised and weighed, subsequently fixed in 10% neutral buffered formalin, embedded in paraffin, and cut into 5 μm sections. Masson’s trichrome staining was used to observe tissue fibrosis according to protocol. The blue-stained collagen and red counterstained muscle were analyzed utilizing ImageJ (Fiji) software. Ten randomly chosen areas at ×50 optical magnification in representative portions of each slide were calculated in a blinded fashion with a square micrometer and the mean area was expressed as the relative percent. The mean percent collagen area was defined according to the formula: collagen area/total visual area × 100%. We and other teams all have previously published research articles using these methods (Gao et al., 2021). The percentage area was selected in the program and generated automatically for each image. The averages were then calculated for each group. For immunohistochemistry, paraffin sections were processed with deparaffinization, antigen retrieval, removal of endogenous catalase, and blockage of the unspecific binding site. Sections were then incubated with primary antibodies overnight at 4°C. After washing in PBS, anti-mouse AF594 (A11032) and anti-rabbit AF-488 (A21206) from Invitrogen were used for incubation for 1 h in the dark at room temperature. Finally, nuclei were counterstained with DAPI. The intensities of α-SMA, Col1, and Fn were obtained using ImageJ software and normalized against DAPI intensities.

### Cell culture and reagents

hBSMCs (No. 4310, ScienCell, San Diego, CA) were cultured with a special smooth muscle cell medium (SMCM) containing 10% FBS and 1% penicillin/streptomycin. Cells between passages 2 and 6 were incubated in conventional culture conditions (5% CO_2_ and 37°C) for all experiments. hBSMCs were pretreated with the indicated intervention reagents for 1 h before exposure to HP. The survivin inhibitor YM155(HY-10194) was obtained from MCE and autophagy antagonist 3-methyladenine (3-MA; M9281) was obtained from Sigma-Aldrich (St. Louis, MO).

### Survivin siRNA transfection

Survivin siRNA and control siRNA were designed and constructed by GenePharma (Shanghai, China) with sequence (forward 5′-GCA​UCU​CUA​CAU​UCA​AGA​A-3′ and reverse 5′-UUC​UUG​AAU​GUA​GAG​AUG​C-3′) were for survivin and sequence (forward 5′-UUC​UCC​GAA​CGU​GUC​ACG​U-3′ and reverse 5′-ACG​UGA​CAC​GUU​CGG​AGA​A-3′) were for control. They were transfected into hBSMCs by Lipo3000 according to the manufacturer’s protocol (Invitrogen). The efficiency of siRNA was detected 48 h after the transfection by Western blot.

### Hydrostatic pressure

hBSMCs were subjected to Hydrostatic pressure (HP) in our designed apparatus, which provided conventional culture conditions (5% CO_2_ and 37°C) for cell growth. Similar to the previous report study, hBSMCs in the apparatus were subjected to HP of 200 cm H_2_O for the pathological parameter mimicking the pathological condition of BOO (Chen et al., 2020a).

### Western blot

Western blot (WB) procedures were as previously described (Chen et al., 2020b), the membranes were incubated overnight at 4°C with the following antibodies: Microtubule-associated protein 1 light chain 3 beta (LC3B) (ab48394; 1:1,000; 17 kDa and 19 kDa), Beclin1 (ab207612; 1:2000; 52 kDa), Survivin (ab134170; 1:1,000; 16 kDa), GAPDH (ab9485; 1:2,500; 37 kDa),Col1 (ab96723; 1:1,000; 129 kDa), Fn(ab268020; 1:1,000; 262 kDa), and PCNA(ab29; 1:1,000; 29 kDa) from Abcam (Cambridge, MA, United States). The membranes were then exposed to an immobilon chemiluminescent substrate.

### 5-ethynyl-2′-deoxyuridine staining

hBSMCs proliferation was also evaluated using the 5-ethynyl-2′-deoxyuridine (EdU) Kit (C10310-1, RiboBio, Guangzhou, China) according to the manufacturer’s instructions. Cells, stained with red, represented proliferation cells, while cell nuclei were blue. The positive cells were analyzed by ImageJ.

### Microarray data of the obstructed bladder

Microarray analysis (service provided by Kangchen Biotech, Shanghai, China) was based on our previous study to evaluate the bladder gene expression in the BOO model and sham-operated group using a Whole Rat Genome Oligo Microarray (Agilent Technologies, Santa Clara, CA) (Yang et al., 2018). After the microarray data of the BOO and sham-operated rats were obtained, we transformed the probe identification numbers into gene symbols. Moreover, we normalized the gene expression values with the Affy package, and log2 transformation and normalization were applied in the Robust Multichip Average signal intensity analysis. Our previous study predicted the potential role of survivin during BOO fibrosis by bioinformatics analyses. To investigate the specificity of survivin in BOO bladder, we further compared all IAP family member’s expression both in mRNA level and protein level between BOO bladder and sham-operated bladder, and we finally confirmed that only survivin expression significantly increased in BOO bladder compared with sham-operated bladder.

### Statistical analysis

Three independent observations for each *in vitro* cellular experiment have been performed (*n* = 3) and *in vivo* rat experiments were divided into three groups (*n* = 8). Statistical analyses were performed with Graph Pad Prism 8 and with SPSS 20.0 software. The data were shown as the mean ± SD. D’Agostino-Pearson normality test was used to evaluate whether the continuous data were normally distributed, and according to the results, Student’s *t*-test or ANOVA for normally distributed data or a Kruskal-Wallis 1-way ANOVA test for not normally distributed data was used. A *p*-value less than 0.05 was considered statistically significant.

## Results

### Bladder outlet obstruction-induced the upregulation of survivin expression

The underlying mechanism of bladder fibrosis flowed by BOO was not well known. Our microarray analysis results showed that among the common IAP members in the bladder, BIRC3 and survivin (BIRC5) were prominently upregulated in the BOO rat bladder when compared with those in the sham-operated bladder, while others were not changed significantly (Figure 1A). However, to better understand the role of survivin in bladder smooth muscle, the bladder-removed mucosa was used to assess the protein expression of survivin and BIRC3 by Western blot. As shown in Figure 1B, the survivin expression of mucosa-denuded bladders in BOO bladder was significantly increased when compared with sham-operated bladder. However, there was no significant difference in BIRC3 protein expression between the sham-operated group and the BOO group.

**FIGURE 1:** BOO-induced upregulation of survivin expression. **(A)** Microarray analysis of the IAP family members in the bladder between BOO group and sham-operated group. **(B)** The protein level of Survivin and BIRC3 in the bladder wall of sham-operated group and BOO group (*n* = 8). Data are presented as the mean ± SD, **p < 0.01; *p < 0.05; (Student’s *t-*test).

### The effect of YM155 on bladder histology alteration secondary to bladder outlet obstruction

Our previous study has predicted that survivin was a critical hub gene in bladder fibrosis (Di et al., 2022). To investigate the effect of survivin during bladder remodeling, the rats were administered survivin inhibitor YM155. Based on the results of urodynamic parameters and Masson staining, BOO was successfully established after obstruction for 6 weeks. As we know, BOO significantly induced the deposition of ECM. After the performance of urodynamic testing, bladders were harvested for the evaluation of bladder weight, histological alteration, and collagen deposition. The results showed that the bladder weights of BOO significantly increased compared with the sham-operated group and the increase was attenuated by the treatment with YM155 (Figure 2A). Nevertheless, body weight did not display evident changes (Figure 2B). We observed the survivin protein in the BOO bladder decreased after the treatment with YM155. Similar trends were observed in the protein levels of PCNA (Figure 2C). Based on Masson’s trichrome staining results, BOO markedly increased the percentage of collagen in the bladder, while treatment with YM155 decreased the percentage of collagen (Figure 2D). As we know, bladder remodeling characterized ECM deposition mainly including Col1 and Fn. As Figure 2E showed, we further found that YM155 mainly decreased the Col1 and Fn of the bladder by the immunohistochemical evaluation (Figures 2F,G). These results indicated that YM155 might reverse bladder remodeling secondary to BOO.

**FIGURE 2:** The effect of YM155 on bladder histology alteration secondary to BOO. **(A)** The alteration of bladder weights. **(B)** The alteration of body weights. **(C)** The protein level of survivin and PCNA in the bladder wall. **(D)**Masson’s trichrome staining of the bladder wall and percent collagen area of the bladder wall. **(E)** The relative expression of Col1 and Fn was obtained by measuring the densities of fluorescence. **(F)** Coimmunostaining of Col1 (green) and *α*-SMA (red) in bladder wall. **(G)** Coimmunostaining of Fn (green) and *α*-SMA (red) in the bladder wall. The staining images were taken under the original magnification ×100. Data are presented as the mean ± SD, *n* = 8. **p < 0.01; *p < 0.05*;* (ANOVA). Scale bar: 200 μm.

### The effect of YM155 on bladder outlet obstruction-induced bladder dysfunction

The bladder function was analyzed according to the urodynamic curve. As shown in Figures 3A–C, the micturition interval in the BOO group was significantly shorter than in the sham-operated group, while treatment with YM155 attenuated the alteration. Micturition pressure, baseline pressure, and threshold pressure were higher in the BOO group compared with the sham-operated group. Baseline pressure was a slight, but significant, increase in BOO treated with YM155 compared with the BOO group, while micturition pressure and threshold pressure have no significant alteration by treatment with YM155 (Figures 3D–G). These observations indicated that the YM155 markedly suppressed the dysuria associated with BOO.

**FIGURE 3:** The effect of YM155 on BOO-induced bladder dysfunction. **(A)** The urodynamic curve of sham-operated rats. **(B)** The urodynamic curve of BOO rats. **(C)** The urodynamic curve of BOO rats that were administered with YM155. **(D)** Baseline pressure, **(E)** micturition pressure, **(F)** threshold pressure, and **(G)** micturition interval in the three groups. Data are presented as the mean ± SD, *n* = 8. **p < 0.01; *p < 0.05; (ANOVA).

### The upregulated survivin enhanced the collagen expression and cell proliferation of hBSMC

As our previous study demonstrated, pressure at 200 cm H_2_O was selected as the optimal pathological parameter mimicking the BOO cell model *in vitro* (Chen et al., 2020a, Jin et al., 2020; Gao et al., 2021). Exposure to 200 cm H_2_O HP for 24 h increased the expression of collagen including Col1 and Fn protein levels. In addition, the analysis of EdU and PCNA expression levels showed that HP enhanced the proliferation as well as upregulated survivin. To explore whether the HP-increased survivin was necessary for fibrosis, hBSMCs were transfected with siRNA before exposure to HP. We first confirmed the successful knockdown of siRNA by the western blot (Figure 4A). As the results of WB showed, survivin siRNA significantly suppressed the HP-induced Col1 and Fn expression (Figures 4B,C). As the results of EdU and the PCNA expression showed, survivin siRNA repressed the HP-induced cell proliferation (Figures 4C,D).

**FIGURE 4:** The pathological pressure-upregulated survivin enhanced the collagen expression and cell proliferation of hBSMC. **(A)** Knockdown of survivin protein by siRNA survivin. **(B)** hBSMC exposure to 200 cm H_2_O for 24 h increased the expression of collagen accompanied by the upregulation of survivin protein, while knockdown of survivin attenuated these changes. **(C)** Knockdown of survivin suppressed the PCNA expression induced by HP. **(D)** EdU assay was used to determine the proliferation of hBSMCs (*n* = 3). **p < 0.01; *p < 0.05; (Kruskal-Wallis 1-way ANOVA). Scale bar: 50 μm.

### Hydrostatic pressure-increased survivin leads to proliferative and fibrotic response through autophagy

Our previous study has demonstrated that autophagy was strongly involved in the function of hBSMCs under HP (Chen et al., 2020b). The emerging data point to several aspects of autophagy that was closely related to survivin protein. To understand whether and how survivin affected autophagy during BOO, autophagy markers in BOO bladder were detected after the treatment with YM155 *in vivo*. We observed the YM155 alleviated BOO-decreased LC3B II/I and Beclin1 (Figure 5A). Cells were exposed to HP, and the level of LC3B II/I and Beclin1 were measured after the treatment with siRNA survivin in the presence or absence of 3-MA. As shown in Figure 5B, siRNA survivin treatment promoted autophagy level, which was evidenced by increased LC3B II and Beclin1, suggesting survivin negatively regulated autophagy level under HP. To investigate whether the increase LC3B II was due to enhanced autophagy or blockage of the lysosomal degradation of autophagic vacuoles, autophagic flux was assessed using the GFP-mRFP-LC3B assay. The results showed that the amounts of autophagosomes and autolysosomes were both increased, indicating that autophagic flux was unobstructed (Figure 5C). We further found that the autophagy inhibitor, 3-MA, not only decreased the siRNA survivin-increased autophagy level but also increased the siRNA survivin-decreased Col1 and Fn (Figure 5D). The PCNA expression and EdU analysis also demonstrated that 3-MA ameliorated the siRNA survivin-increased proliferation (Figures 5D,E). These results suggested that survivin negatively regulated autophagy, which played a critical role in fibrosis and proliferation of hBSMCs.

**FIGURE 5:** Increased survivin by HP led to proliferative and fibrotic response through autophagy. **(A)** YM155 increased the autophagy markers of the BOO bladder wall (*n* = 8). **(B)** siRNA survivin attenuated the decreased autophagy of hBSMCs induced by HP, which was evidenced by increased LC3B II and beclin1 (*n* = 3). **(C)** GFP-mRFP-LC3B assay evaluated whether autophagic flux was unobstructed. **(D)** 3-MA decreased the siRNA survivin-increased autophagy level as well as the siRNA survivin-decreased Col1, Fn, and PCNA expression (*n* = 3). **(E)** EdU assay was used to determine the proliferation of hBSMCs (*n* = 3). Data are presented as the mean ± SD, **p < 0.01; *p < 0.05; [ANOVA for **(A)**; Kruskal-Wallis 1-way ANOVA for **(B–E)**]. Scale bar: 20 μm for **(C)** and 50 μm for **(E)**.

## Discussion

Accumulating evidence suggests that the impairment of bladder morphology and bladder function secondary to BOO is associated with fibrosis, which is characterized by bladder smooth muscle hypertrophy and ECM deposition (Uvelius, Persson, and Mattiasson 1984; Metcalfe et al., 2010; Metcalfe et al., 2010). There is widespread consensus that ECM deposition in the detrusor layer is the primary reason for dysfunction. Understanding the underlying mechanism from obstruction to hypertrophy and fibrosis using rat models may contribute to identifying targets for pharmaceutical intervention at the appropriate stage of bladder remodeling.

Emerging studies indicate that survivin is critically involved in various physiological and pathological processes, such as wound healing, neovascularization, scar formation process, and so on, due to its dual effects of promoting the cell cycle and inhibiting apoptosis (Ding et al., 2015; Miyamoto et al., 2021; Sharma et al., 2021). Our previous report predicted that survivin was well related to bladder fibrosis by bioinformatics analyses from the whole bladder. To better understand the role of survivin in bladder smooth muscle, the bladder wall tested in the present study was removed mucosa. We demonstrated that among IAP members, BIRC3 and survivin were prominently upregulated. Based on the potential role in bladder fibrosis, it was of great interest to explore the effect of survivin on the pathological process of BOO. Altered ECM composition, especially, Col1 and Fn, has been reported in the hypertrophic bladder during the fibrotic stage of hypertrophy. The result showed that targeting inhibition of survivin by YM155 could downregulate the ECM deposition and improve bladder dysfunction secondary to BOO.

The bladder detrusor, which is mainly composed of smooth muscle cells, is considered to be the important structural unit of the bladder wall. The late stage of BOO is characterized by muscle hypertrophy and enhanced production of extracellular matrix constituents. Besides the BSMC secreted collagens, other mechanisms such as epithelial-mesenchymal transition (EMT), fibroblast-to-myofibroblast transition (FMT), and macrophage-myofibroblast transition (MMT) are all involved in bladder fibrosis. Although collagen that existed in the bladder detrusor is not the most, the collagens in intercellular spaces of smooth muscle cells seriously affect bladder function. The biomechanical force caused by BOO is a critical element for bladder smooth muscle cell function and phenotype. Therefore, the present study focused on the bladder smooth muscle cells. The persistent obstruction increased intravesical pressures, which played a critical role in bladder remodeling (Chen et al., 2012; Liang et al., 2017). To extensively illustrate the underlying mechanism, hBSMCs were exposed to the HP of 200 cm H_2_O mimicking the conditions of BOO, and were used as the experimental model for the present investigation. We found that HP of 200 cm H_2_O significantly increased collagen expression and enhanced cell proliferation as well as upregulated survivin, which was similar to the results *in vivo*. We further used siRNA to knock down survivin protein, the results showed that siRNA survivin ameliorated the HP-increased fibrotic and proliferative response.

As a multifunctional factor widely existing in mammals, autophagy participates in various physiological and pathological processes, such as immunity, inflammation, fibrosis, and so on. Our previous study indicated that HP significantly enhanced the proliferation and contraction of BSMCs, and we found that autophagy was of importance to BSMCs dysfunction. While the underlying mechanism is not well known. Emerging evidence suggests that crosstalk between apoptosis and autophagy plays an important role in supporting cell survival and proliferation. Survivin, as a member of the IAP family, was initially thought to be a connection with autophagy. We firstly indicated that survivin knockdown abolished the HP-decreased autophagy level by assessing the LC3B II/I ratio and Beclin1 expression. Subsequent experiments further revealed that autophagy inhibitor 3-MA suppressed the survivin knockdown-induced changes.

This present study still has some limitations. Firstly, our study failed to explore human BOO tissues or samples for ethical reasons. Secondly, the effect of YM155 on HP-induced fibrosis of hBSMCs needs to be further explored. In conclusion, HP-induced survivin negatively regulated autophagy, which played a critical role in the pro-fibrosis and pro-proliferative of hBSMCs *in vitro*. A novel anti-fibrotic and anti-proliferative function of survivin might represent a potential target for therapeutic strategies in bladder remodeling. Clinical trials were needed to validate the effect of survivin on bladder dysfunction and bladder fibrosis in the future.

## Data Availability

The original contributions presented in the study are included in the article/supplementary material, further inquiries can be directed to the corresponding authors.
